This article has been retracted.

# Effect of Orthodontic Treatment on Anterior Tooth Displacement in Patients with Periodontal Disease: A Meta-Analysis

**DOI:** 10.1155/2021/8761215

**Published:** 2021-10-31

**Authors:** Jia Hou, Yunzhu Qian, Guowu Ma, Huan Gao, Jianxin Yang, Jianlin Fan

**Affiliations:** Department of Stomatology, The Second Affiliated Hospital of Soochow University, 1055 Sanxiang Road, Suzhou City, Jiangsu Province 215004, China

## Abstract

**Objective:**

To systematically evaluate the effect of orthodontic treatment (ODT) on anterior tooth displacement (ATD) in patients with periodontal disease.

**Methods:**

PubMed, Web of Science, Embase, China National Knowledge Infrastructure, and Wanfang databases were electronically searched for relevant literature studies on ODT and basic treatment for ATD in patients with periodontal disease, and then the related journals and reference lists of the included studies were manually searched. The search time was set from January 2010 to May 2021. Stata 16.0 software was used for meta-analysis.

**Results:**

Totally, 783 articles were retrieved, and finally, 14 studies were included. The effective rate of basic treatment combined with OTD was significantly higher than that of basic treatment alone (OR = 7.27, 95% CI: 3.76, 14.04). Specifically, the combined treatment led to lower values of periodontal pocket depth (SMD = −2.30, 95% CI: −2.94, −1.66), anterior overjet (SMD = −2.75, 95% CI: −3.72, −1.78), anterior overbite (SMD = −2.13, 95% CI: −3.16, −1.10), and periodontal bleeding index (SMD = −4.25, 95% CI: −5.48, −3.03) compared with those of basic treatment alone.

**Conclusion:**

Compared with basic treatment, ODT combined with basic treatment is more effective for patients with periodontal disease-caused ATD and can also improve the clinical symptoms of patients.

## 1. Introduction

Periodontal disease, a worldwide disease with a high prevalence and incidence, is common in patients with oral-related diseases [1]. Its incidence rises with age, and it is estimated that more than 90% of the general population suffers from periodontal disease [2]. In case of no prompt treatment, periodontal disease may cause a variety of diseases. According to clinical observations, periodontal disease can lead to the loss of supporting structures. When periodontal disease causes damage to the supporting structures that maintain the physiological position of the teeth, patients may experience pathological tooth displacement, such as forward tilting forward anteversion, diastemata, rotation, extrusion, migration, and even tooth loss [3]. Periodontitis with advancement of the incisors leads to premature occlusal contact and accelerates the loss of periodontal support structures, thus negatively affecting tooth esthetics and hindering occlusion in daily life [4, 5].

The primary current treatment approaches to periodontal disease are conventional periodontal therapy, medical therapy, surgery, and periodontal tissue regeneration [6]. Orthodontic treatment (ODT) is most commonly used clinically for patients with anterior tooth displacement (ATD), enhancing appearance and function of teeth by correcting or moving them [5]. In clinical practice, ODT focuses on adjusting the coordination between facial bones, teeth, and facial nerves and muscles in the maxillofacial region through various orthodontic appliances. The ultimate orthodontic goal is to achieve balance, stability, and esthetics of the stomatognathic system [7]. Studies have shown that ODT can help maintain the health of the teeth, gingiva, and temporomandibular joint, but there is limited evidence and no systematic evaluation on the therapeutic effect of ODT on ATD caused by periodontal disease [8]. Hence, by using meta-analysis, this study comprehensively and systematically assessed the efficacy of ODT for periodontal disease-caused ATD, thereby providing a reference for its clinical treatment and prognostic evaluation.

## 2. Materials and Methods

The systematic review was conducted in accordance with the guidelines outlined in the Preferred Reporting Items for Systematic Reviews and Meta-Analyses (PRISMA) statement [9].

### 2.1. Literature Retrieval

PubMed, Web of Science, Embase, China National Knowledge Infrastructure, and Wanfang Data were searched for relevant English and Chinese articles published from January 2010 to May 2021. The keywords were preliminarily set as follows: “Orthodontic treatment” and “Periodontal disease” or “Anterior tooth displacement” or “Periodontitis.”

### 2.2. Inclusion Criteria Based on PICOS

  Population: patients with indications for ODT by imaging and oral routine examination and with periodontal disease-caused ATD.
  Intervention: the control group received basic treatment for periodontal disease, mainly including cleaning the oral periodontal, repairing the periodontal root surface, removing the oral lesions, and controlling the condition by antibiotic treatment; the treatment group received basic treatment combined with ODT using a straight wire arch correction technique with titanium-nickel wires.
  Comparators: participants in basic treatment and orthodontic treatment.
  Outcome: treatment response rate, periodontal pocket depth, anterior overjet, anterior overbite, and periodontal bleeding index. All of these outcome measures were assessed more than 6 months after treatment. Effective treatment referred to basic restoration of normal anterior function and normal tooth esthetics, basic elimination of periodontitis symptoms, and improved tooth mobility after treatment. Ineffective treatment referred to that the effective indicators cannot be met after treatment; patients showed no significant changes in the anterior tooth function and could not chew, with tooth mobility and presence of periodontitis symptoms.
  Studies: randomized controlled trial, clinical controlled trial, and cohort study.

### 2.3. Exclusion Criteria

The exclusion criteria were as follows: (1) literature without data required by this meta-analysis or access to obtain the original text; (2) low-quality literature, literature with missing data, and repeated reports; (3) literature on ATD that was not caused by periodontal disease; (4) case reports, systematic reviews, and animal experiments.

### 2.4. Data Extraction

Two investigators independently completed the literature screening and data extraction. Specifically, after excluding the literature that obviously did not meet the screening criteria, the remains were selected by reading titles and abstracts and even full text and cross-checked to identify the final included articles. During this process, any disagreement was resolved through discussion between the two investigators or through third-party assistance. The following data were extracted: name of the first author, year of publication, study site, study design, and main outcome measures.

### 2.5. Statistical Analyses

Statistical analysis was performed by using Stata 16.0 software (StataCorp, College Station, TX, USA). Outcome measures were expressed as standardized mean difference (SMD) or odds ratio (OR). Heterogeneity among the studies was assessed using the *I*^2^ statistic. In case of homogeneity (*P* > 0.1, *I*^2^ < 50%), the fixed-effect model was used for meta-analysis; otherwise, the random-effect model was applied. Moreover, sensitivity analysis was adopted for testing the stability of the overall result. If more than 10 studies were included, funnel plots were used to assess publication bias.

## 3. Results

### 3.1. Basic Characteristics of Included Articles

The initial retrieval yielded 783 relevant articles, and then 257 duplicated articles were removed. Next, 367 irrelevant articles were excluded based on titles or abstracts, and 145 articles were further excluded by reading full text. Fourteen articles were finally included for meta-analysis [10–23]. The specific literature screening process is shown in Figure 1, and the basic characteristics of the included ones are shown in Table 1.

### 3.2. Comparison of Treatment Response Rate between the Two Groups

Ten articles compared the treatment response rate between the two groups [10, 14, 16, 18, 20, 23]. No significant heterogeneity among the studies was observed (*I*^2^ = 0.0%, *P*=0.999), so the fixed-effect model was utilized for analysis. Meta-analysis showed a higher response rate in the treatment group compared with the control group (OR = 7.27, 95% CI: 3.76, 14.04) (Figure 2(a)). In addition, the funnel plot in a symmetrical manner suggested that the possibility of publication bias in the included literature was small (Figure 2(b)). In sensitivity analysis, the 10 studies were eliminated one by one; the result showed that the pooled effect size was still of a statistical significance, and the forest plot direction did not change significantly before and after removal (Figure 2(c)).

### 3.3. Comparison of Clinical Outcome Measures between the Two Groups

Fourteen articles compared the periodontal pocket depth after treatment between the two groups [10–23]. The random-effect model was used for meta-analysis because of the significant heterogeneity among the studies (*I*^2^ = 93.0%, *P* ≤ 0.001). The pooled result revealed that the periodontal pocket depth of patients in the treatment group was markedly lower than that of the control group after treatment (SMD = −2.30, 95% CI: −2.94, −1.66) (Figure 3(a)).

Thirteen articles compared the anterior overjet after treatment between the two groups [10, 17, 19–23]. With marked heterogeneity among these studies (*I*^2^ = 96.3%, *P* ≤ 0.001), the random-effect model was utilized and subsequently estimated a shorter anterior overjet in the treatment group (SMD = −2.75, 95% CI: −3.72, −1.78) (Figure 3(b)).

Nine articles compared the anterior overbite after treatment between the two groups [14, 16, 18–23]. By using the random-effect model (*I*^2^ = 95.9%, *P* ≤ 0.001), the result suggested that patients in the treatment group had significantly shorter anterior overbite (SMD = −2.13, 95% CI: −3.16, −1.10) (Figure 3(c)).

Twelve articles compared the periodontal bleeding index after treatment between the two groups [10, 13–23]. With the application of the random-effect model (*I*^2^ = 96.6%, *P* ≤ 0.001), the results showed that the periodontal bleeding index showed a lower value in the treatment group (SMD = −4.25, 95% CI: −5.48, −3.03) (Figure 3(d)).

Furthermore, the funnel plot in a symmetrical manner suggested a small possibility of publication bias in the included literature (Figures 4(a)–4(d)). In sensitivity analysis, the studies were eliminated one by one; the result showed that the pooled effect size was still of a statistical significance, and the forest plot direction did not change significantly before and after removal (Figures 5(a)–5(d)).

## 4. Discussion

Gingival inflammation and periodontitis is mainly caused by and aggravated by plaque damage to the tissue structure [8]. And ODT is introduced to a predisposing factor for periodontal disease; for example, orthodontic devices may serve for bacterial accumulation [24]. The massive accumulation of bacteria may further cause the transformation of subgingival plaque into more aggressive pathogen populations, consequently leading to gingivitis into more severe periodontitis [25]. However, before and during ODT, strict cavity cleaning and protection of the tooth gingiva to reduce the bleeding index can significantly reduce the content of oral disease-related bacteria [26]. Additionally, with the conditions of effective plaque control and good periodontal health, orthodontic devices will not cause periodontal damage clinically [27]. However, when the inflammation in the patient's oral cavity is not completely controlled, ODT may trigger inflammation and accelerate periodontal destruction, resulting in further loss of attachment, and even maintaining good oral hygiene during ODT cannot avoid the damage of inflammation to orthodontic teeth [28]. Therefore, inflammation should be controlled in a timely manner before ODT for patients with ATD caused by periodontal disease. In the present study, we found that ODT in combination with basic treatment can significantly increase the treatment efficiency, achieving inflammatory control and orthodontics.

According to the relevant meta-analysis, orthodontic appliances will not lead to clinically significant irreversible periodontal tissue destruction [29]. For adults with severe periodontal disease, there will be no situation where ODT cannot be used. In the results of this study, ODT combined with basic treatment significantly improved the periodontal pocket depth, anterior overjet, anterior overbite, and bleeding index of patients. In the previous studies, periodontal disease was likely to lead to the deterioration of dentition, including the deterioration of peripheral pocket depth, overjet, bleeding index, and other conditions [30]. Compared with patients with normal periodontal support, patients with reduced periodontal tissue due to periodontal disease show a reduction in the stressed periodontal ligament surface and different biological and biomechanical conditions from normal teeth. In periodontally compromised teeth, the center of resistance moves apically with the anatomy of the periodontal tissue, which leads to an increase in the extrusion component of the applied force and greater moments during the application of force [31]. Therefore, it is particularly vital to control the tooth position, especially in the vertical direction. Some studies have pointed out that ODT is associated with an improvement of the pocket probing depth and crown-root ratio of patients [32]. In addition, ATD can cause thin soft tissue or bone dehiscence in specific cases, involving areas with low resistance to inflammation or trauma and thus leading to higher inflammation rate of the areas. Hence, orthodontic tooth movement should be preceded by surgery to increase the thickness of the periodontal tissue; otherwise, it easily leads to bone dehiscence [33]. It has also been stated that the compressed elastic gingiva is the reason for the posttreatment recurrence of ATD [34]. However, this study found that ODT combined with basic treatment had a better therapeutic effect than that of basic treatment alone. Collectively, periodontal disease-caused ATD is a complex condition, but ODT combined with basic treatment can significantly improve the treatment efficiency and achieve a good therapeutic effect.

This meta-analysis has some limitations. (1) Only 14 studies were included, and the sample size of each trial was small, which affected the final results; (2) all patients were from China, based on clinical randomized controlled trials, and the quality of the comprehensive evaluation literature was not very high; (3) due to the limitation of data sources for the meta-analysis, it was difficult to obtain unpublished data, which had an impact on the results.

## 5. Conclusion

By using meta-analysis, it has been proved that ODT combined with basic treatment can markedly improve periodontal disease-caused ATD, showing higher safety and efficacy than basic treatment alone. However, due to the limitation of the number and quality of included studies, the above conclusions still need to be verified by more high-quality studies.

## Figures and Tables

**Figure 1:** Literature screening process.

**Figure 2:** Forest plot of treatment response rate in the two groups (a); funnel plot of treatment response rate in the two groups (b); sensitivity analysis of treatment response rate in the two groups (c).

**Figure 3:** Forest plots of clinical outcome measures: (a) periodontal pocket depth after treatment; (b) anterior overjet after treatment; (c) anterior overbite after treatment; (d) periodontal bleeding index after treatment.

**Figure 4:** Funnel plots of clinical outcome measures: (a) periodontal pocket depth after treatment; (b) anterior overjet after treatment; (c) anterior overbite after treatment; (d) periodontal bleeding index after treatment.

**Figure 5:** Sensitivity analysis of clinical outcome measures: (a) periodontal pocket depth after treatment; (b) anterior overjet after treatment; (c) anterior overbite after treatment; (d) periodontal bleeding index after treatment.

**Table 1:** The basic characteristics of the included literature.

First author	Year	Sample time	Diagnostic method	Cases (Treat/Con)	Follow-up time (months)	Age (years)		Sex ratio (M : FM)		Study design	Outcome measured
						Treat	Con	Treat	Con		
Huang [10]	2019	2014.12–2017.12	X-rays	44/44	6–12	34–62	32–61	29 : 15	28 : 16	RCT	① + ② + ③ + ④
Jiang [11]	2019	2016.3–2017.3	X-rays	30/30	6–12	23–68	23–68	10 : 20	12 : 18	RCT	① + ② + ③ + ④
Li [12]	2018	2015.11–2017.10	X-rays	25/25	6–12	23–62	22–62	14 : 11	15 : 10	RCT	① + ② + ③ + ④
Li [13]	2019	2016.4–2018.7	X-rays	33/33	6	35.51 ± 4.34	35.63 ± 4.25	18 : 15	19 : 14	RCT	① + ② + ③ + ④
Li [14]	2017	2014.2–2017.2	X-rays	24/24	6–12	35.8 ± 10.6	34.6 ± 10.3	13 : 11	14 : 10	RCT	① + ② + ③ + ④
Liu [15]	2019	2015.6–2018.6	X-rays	40/40	6–12	36.6 ± 9.4	35.6 ± 8.4	20 : 20	22 : 18	RCT	① + ④
Man [16]	2018	2016.12–2018.3	X-rays	41/41	6–12	36.20 ± 2.17	37.51 ± 1.68	23 : 18	22 : 19	RCT	① + ② + ③ + ④
Ning [17]	2018	2016.12–2017.12	X-rays	33/33	6–12	39.66 ± 6.56	38.28 ± 5.56	17 : 16	16 : 17	RCT	① + ② + ③ + ④
Wang [18]	2019	2015.1–2019.1	X-rays	29/29	6–12	40.26 ± 0.45	40.84 ± 0.41	18 : 11	16 : 13	RCT	① + ② + ③ + ④
Xiao [19]	2016	2013.1–2016.1	X-rays	30/30	6–12	41.85 ± 3.76	41.62 ± 3.94	19 : 11	20 : 10	RCT	① + ② + ④
Yang [20]	2018	2016.5–2018.5	X-rays	36/36	6–12	35.1 ± 3.4	34.4 ± 2.8	21 : 15	20 : 16	RCT	① + ②
Zhang [21]	2019	2016.1–2019.1	X-rays	32/32	6–12	42.9 ± 2.7	43.4 ± 2.5	13 : 19	14 : 18	RCT	① + ②
Zhang [22]	2020	2017.1–2019.7	X-rays	24/24	6–12	34.21 ± 6.43	34.56 ± 6.78	17 : 7	15 : 9	RCT	① + ② + ③ + ④
Zhou [23]	2018	2017.1–2018.7	X-rays	30/30	6–12	41.85 ± 3.76	41.62 ± 3.94	20 : 10	19 : 11	RCT	① + ② + ④

Treat: treatment group; Con: control group; M: male; FM: female; RCT: randomized controlled trial; ①: depth of the periodontal pocket; ②: anterior overjet; ③: anterior overbite; ④: periodontal bleeding rate.

## Data Availability

The data used to support the findings of this study are available from the corresponding author upon request.
